The article "Path analysis based on genetic association of yield components and insects pest in upland cotton varieties" was retracted in 2022. Reasons: compromised peer review; a conflict of interest; concerns about the authorship.

# Path analysis based on genetic association of yield components and insects pest in upland cotton varieties

**DOI:** 10.1371/journal.pone.0260971

**Published:** 2021-12-30

**Authors:** Mussarat Shaheen, Hafiz Abdul Rauf, Muhammad Ahmed Taj, Muhammad Yousaf Ali, Muhammad Amjad Bashir, Sagheer Atta, Hasnain Farooq, Reem A. Alajmi, Mohamed Hashem, Saad Alamri

**Affiliations:** 1 Cotton Research Institute, Khan pur, Punjab, Pakistan; 2 Rural Health center 222EB, Health department Govt. of Punjab, District Vehari, Pakistan; 3 Research & Education Development Department, Rural Education and Economic Development Society (REEDS) Pakistan, Rahim Yar Khan, Punjab, Pakistan; 4 Department of plant protection faculty of agricultural sciences, Ghazi University, Dera Ghazi Khan, Punjab, Pakistan; 5 Department of Environmental Sciences, University of California, Riverside, CA, United States of America; 6 Department of Forestry, Faculty of Agricultural Sciences, Ghazi University, Dera Ghazi Khan, Pakistan; 7 Zoology Department, College of Science, King Saud University, Riyadh, Saudi Arabi; 8 Department of Biology, College of Science, King Khalid University, Abha, Saudi Arabia; 9 Faculty of Science, Botany and Microbiology Department, Assiut University, Assiut, Egypt; Harran Üniversitesi: Harran Universitesi, TURKEY

## Abstract

*Gossypium hirsutum* L. is also called upland cotton or Mexican cotton. It is the most widely cultivated species of cotton in the whole world. Globally, about 90% of all cotton production comes from the cultivars derived from this species. Some genetic parameters like monopodial branches per plant, sympodial branches per plant, sympodial branch length, bolls per plant, boll weight, sympo-boll distance, Ginning Out Turn%, staple length (rg = 0.9199**), and fiber strength along with seed cotton yield were evaluated for their potential utilization via selection in seed cotton yield improvement. Significant positive genetic correlations were estimated for monopodial branches per plant (rg = 0.9722**), sympodial branches per plant (rg = 0.7098**), sympodial branch length (rg = 0.617**), bolls per plant (rg = 0.8271**), boll weight (rg = 0.8065**), sympo-boll distance (rg = 0.6507**), Ginning Out Turn (GOT)% (rg = 0.7541**), staple length (rg = 0.9199**), and fiber strength (rg = 0.7534**) with seed cotton yield. A path analysis of all the yield traits under study revealed strong positive direct effects of monopodial branch length (1.1556), sympo-boll distance (0.8173) and staple length (0.7633), while plant height exerted a highly strong direct negative effect (-1.2096) on yield. It is concluded that a direct selection based on monopodial branch length and sympo-boll distance, and staple length is effective, whereas, monopodial branch length, and sympodial branch length are good selection indicators via bolls per plant for yield improvement in cotton.

## Introduction

*Gossypium hirsutum* L. also known as upland cotton [1] or Mexican cotton, is the most widely cultivated species of cotton in the world. Globally, ~90% cotton production comes from the cultivars derived from this species. Most commonly short staple cotton is the characteristic of upland cotton. To overcome this scientist are working to get extra-long stapple in upland cotton [2]. Upland cotton is primarily used in making denim jeans as well as flannel cloth [3]. Scientist are working on genetic variations in upland cotton to overcome different issues and challenges like salt tolerance [4], fiber traits [5], resistance against bacterial blight [6] and insect resistance [7]. Presence of different secondary endosymbionts in whitefly also determine the virus infection severity [8]. A part from adoption of water saving techniques like drip irrigation and use of sprinkler systems to cultivate cotton [9] new varieties of upland cotton should be developed through breeding and genetic modification which are drought tolerant. Though whitefly control by use of RNAi against candidate genes is found quite effective [10] some varieties which are tolerant to attack of whitefly should be raised through breeding. Some new varieties which are high yielding and are adopted to severe temperature zone are being introduced like RH-647 [11]. A pleotropic gene effect could embrace a change in one character that is most often accompanied by changes in the expression of several others traits either in same direction or antagonistic way; therefore, deriving a basic knowledge of genetic perspectives of various traits, magnitude and direction of reciprocal genetic association is very important [12, 13]. Cotton breeders forfeit great efforts and breeding approaches through illustrating genetic basis of gene mechanism, inherited association of either individual per collaborative impact of various agronomic and economic traits for genetic manipulations in breeding population [14]. Practically, simple correlation does not explain the causes, origin and pathway of interrelationship of genetic parameters for depiction of effective selection parameters for evaluation of breeding material [15, 16]. Seed cotton yield is polygenic and highly intricate trait for improvement is under collaborative impact of various quantitative characters association hence, a path coefficient analysis helps to measure and engrave the direct and indirect effects of various component traits for decisive evaluation of yield component contribution to economic yield [13, 17, 18].

Several cotton breeders previously worked out the direct and indirect effect of various plant traits in yield improvement. Genetic correlations of various economic traits with yield and reported positive and significant genotypic correlation of staple length, lint% and fiber fineness with yield and strong direct effects of lint%, staple length and fiber fineness on yield were estimated [19]. In 2004 significant positive genetic correlation of boll per plant with seed cotton yield and direct contribution bolls per plant and sympodial branches per plant manifested maximum positive direct effect on seed cotton yield were estimated [20]. Highly significant positive correlation of boll weight, boll per plant, plant height and seed index with seed cotton yield and maximum direct effect of boll weight and seed index to yield were also reported [21]. Another study revealed a positive and highly significant correlation of sympodial branches per plant, boll per plant, boll weight, plant height and yield [22]. Genetic correlations and path coefficient analysis for seed oil, yield and fiber quality traits in *Gossypium hirsutum* L were studied and revealed positive significant correlation with number of sympodial branches per plants, bolls per plant, boll weight and GOT % with yield and estimated a positive direct effect exerted by boll weight and sympodial branches per plant on seed cotton yield [23]. The significant positive correlation positive direct effect of sympodial branches per plant, bolls per plant and boll weight and negative correlation of monopodial branches per plant with seed cotton yield was reported in 2010 [15]. Moreover, it was suggested that monopodial branches per plant, sympodial branches per plant, bolls per plant and boll weight as good indicators of effective selection in cotton breeding programs. In correlations and path analysis of fifteen genotypes and six upland cotton traits, Salahuddin *et al*., 2010 reported positive correlation of sympodial branches per plant, bolls per plant, boll weight, GOT % and lint index to yield and strong positive direct effect of bolls per plant and boll weight on seed cotton yield. Positive significant correlation of bolls per plant, sympodial branches per plant, plant height, lint index and boll weight to yield was also studied [24]. Positive correlation and maximum direct effects of sympodial

## Materials and methods

### Experiment location

The study was conducted in experimental area of Cotton Research Institute, Khanpur, Punjab, Pakistan. The overall climatic conditions of this area are hot severe summer and dry atmosphere.

### Experiment design

Experiment was conducted according to Randomized Complete Block Design (RCBD) with three replications. A total 34 genotypes of a breeding population were grown in field conditions by two successive years of 2019 and 2020. Each Plot area was 28 × 10 ft^2^ separated with a path of 5ft were sown at beds with R×R distance and P× P distance of 9 inch throughout season maintaining of all the recommended agronomic practices of fertilizer application, irrigation and crop protection measures that were followed from sowing till maturity and harvesting. On harvesting of mature crop data were recorded in each entry for 25 randomly selected plants on crop maturity for recording of data and agronomic data for monopodial branches per plant (MBP), monopodial branch length (MBL), sympodial branches per plant (SBP), sympodial branch length (SBL), sympo-boll distance, (SBD), bolls per plant (BP) Plant height and 50 Boll weight. Means were computed in each replication for each entry. The seed cotton samples of 50 bolls of all the plants in each entry were subjected to ginning by a single roller electrical gin in the laboratory on individual plant basis. After ginning of 50g seed-cotton, ginning out turn (GOT) % of samples were estimated. Lint samples were subjected to further fiber traits like staple length (SL), fiber strength (tpsi), (FS) and fiber fineness (FF) micronaire by using spinlab ® HVI-900 at Cotton Research Station (CRS) Multan, Pakistan. Means of the replicated form of recorded data computed simply generating in Microsoft Office® 2007. Phenotypic correlations among traits were calculated from mean values and genetic variance was obtained from the combined analysis of variance for each replication. The genetic and phenotypic components of correlation were determined to establish the association among all the characters *vis a vis* to seed cotton yield as shown in (Table 2). The genetic correlations were further subjected to derive direct, residual and indirect influence of each character towards plant yield as shown in (Table 3).

## Results

Analysis of Variance (ANOVA) revealed highly significant differences *p≤0*.*01* and p≤0.05 for monopodial branches per plant; monopodial length, sympodial branches per plant, sympodial length, plant height, bolls per plant, boll weight, sympo-boll distance, GOT%, fiber finesse, fiber strength and finally yield were evaluated for significant variations exist among the genotypes of breeding population as shown in (Table 1).

**Table 1:** Estimates of genetic variability from Analysis of Variance (ANOVA).

SOV	df	MBP	MBL (cm)	SBP	SBL (cm)	PH (cm)	BP	BW (g)	SBD (cm)	GOT %	SL (cm)	FF (mic)	FS (g per tex)	Yield (Kg)
**∑δ** ^**2**^ **Replication**	2	0.030	1581.7	1.757	131.453	5288.21	66.19	0.057	0.031	1.488	1.533	10.715	0.172	132.93
**∑δ** ^**2**^ **Genotypes**	33	14.03	2244.8	112.85	532.316	12531.40	3183.68	15.90	9.99	457.67	215.58	1002.96	5.55	14577.5
**∑δ** ^**2**^ **Error**	67	7.83	3493.9	159.24	987.47	10681.06	3510.83	5.11	5.43	117.09	94.48	750.84	8.03	10538
**Total**	102	21.89	7320.5	273.85	1651.24	28500.68	6760.71	21.07	15.46	576.26	311.59	1764.52	13.76	25248.4
**S.D**	-	0.46	8.514	1.647	4.04	16.79	8.18	0.45	0.39	2.38	1.75	4.18	0.36	15.81
**S.E**	-	0.04	0.843	0.163	0.40	1.66	0.81	0.045	0.039	0.237	0.174	0.41	0.037	1.56
**CV%**	-	23.24	9.96	8.11	20.25	11.58	18.98	9.78	12.63	3.53	4.42	9.24	6.73	8.69

df = degree of freedom, MS = Mean squares, SOV = Source of variation, ∑δ^2^ = sum of squares. S.D = standard deviation, S.E = standard error, CV% coefficient of variation.

### Coefficients of genetic correlations

The estimated phenotypic correlation coefficients were comparatively lower in magnitude than genotypic correlation for their corresponding coefficients of correlation. Monopodial branches per plant was strongly and significantly correlated with monopodial branch length as (rg = 0.94**), bolls per plant (0.67**) with yield (rg = 0.97**), while it was strongly negatively correlated with GOT% (rg = —0.80**), fiber strength (rg = —0.73**), and moderately with plant height (rg = -0.39). Negligible association with all other characters were reported in the current study (Table 2). Monopodial branch length was estimated to be positively correlated with plant height as (rg = 0.33) and cotton yield as (rg = 0.22) and moderate negative association of the character with number of bolls per plant (rg = -0.27) as shown in Table 2. Sympodial branches per plant was estimated to impend a positive genetic association with other economic traits like sympodial branch length (rg = 0.39), bolls per plant (rg = 0.54) and seed cotton yield as (rg = 0.70**), while highly significant negative genetic correlation plant height as (rg = -0.65), and fiber strength was (rg = —0.9.10**), while exhibited a negligible association with all other characters under investigation as shown in (Table 2). Sympodial branch length exhibit positive moderate genetic correlation with plant height was (rg = 0.27), fiber strength as (rg = 0.28), and significant positive correlation with bolls per plant (rg = 0.59), and seed cotton yield as (rg = 0.61**), whereas negligible association with all other characters under investigation as shown in (Table 2). As far as plant height and traits are concerned it exhibited negligible and genetic associations with all traits understudy and finally bolls per plant exerted a positive correlation with seed cotton yield (rg = 0.82**) as shown in (Table 2). The boll weight was estimated to exhibit a positive association with sympo-boll distance as (rg = 0.261), with GOT% as (rg = 0.29), staple length (rg = 0.35*). Finally, it possessed significant positive correlation with seed cotton yield as (rg = 0.80**), while a significant negative association of boll weight with fiber strength (rg = 0.68**) as shown in (Table 2). Sympo-boll distance exerted moderate positive correlation with GOT % (rg = 0.27), and highly significant positive association with yield as (rg = 0.65**), and strong negative association with fiber strength (rg = -0.53**) as shown in (Table 2). As far as GOT% exhibit a strong positive association to seed cotton yield as (rg = 0.75**) and significant negative association of the character under inference with fiber strength as (rg = -0.44*) shown in (Table 2). Staple length has been estimated for strong positive genetic correlation with fiber strength as (rg = 0.75**) and seed cotton yield as (rg = 0.91**). Whereas, fiber finesse has moderate negative genetic correlation to seed cotton yield (rg = -0.26) and negligible association with fiber strength as shown in (Table 2) and fiber strength was estimated to be significantly and strongly associated to seed cotton yield (rg = 0.87**) is illustrated in (Table 2).

**Table 2:** Estimated genetic and phenotypic coefficients of correlation for various agronomic and fiber traits towards yield of upland cotton.

Variables		MBL (cm)	SBP	SBL (cm)	PH (cm)	BP	BW (g)	SBD (cm)	GOT%	SL (mm)	FF) (mic)	FS (g per tex)	Yield (Kg)
**MBP**	rg	0.94**	0.060	0.19	‒0.39	0.67**	0.042	‒0.00	‒0.80**	‒0.09	‒0.18	‒0.73**	0.97**
	rp	3.93**	0.55	‒1.7	‒4.97	4.31	‒0.02	‒0.03	‒0.75	‒3.21*10^−3^	0.19	‒0.35	‒2.08
**MBL (cm)**	rg		0.01	0.15	0.33*	‒0.27	0.01	0.02	‒0.00	0.06	2.02*10^−3^	0.16	0.22*
	rp		2.332*10^−3^	0.07	0.29	‒0.19	3.81*10^−3^	0.02	‒0.01	0.04	0.18	2.02*10^−3^	‒0.14
**SBP**	rg			0.39*	‒0.65**	0.542**	0.10	0.02	0.01	0.12	0.02	‒0.9.10**	0.70**
	rp			0.72**	‒1.54**	0.075	0.16	‒5.03*10^−4^	0.02	0.05	0.02	‒0.94	2.12
**SBL (cm)**	rg				0.27*	0.59**	0.029	‒0.77*10^−4^	‒0.167	9.91*10^−4^	‒0.63*10^−5^	.28*	0.61**
	rp				0.20	0.41	0.02	‒0.77*10^−4^	‒0.18	9.91*10^−4^	0.29	‒6.31*10^−4^	1.08**
**PH (cm)**	rg					0.09	‒1.385*10^−3^	3.22*10^−3^	‒0.03	0.038	1.61*10^−3^	0.07	‒0.05
	rp					0.09	‒1.384*10^−3^	3.21*10^−3^	‒7.06*10^−3^	2.977*10^−2^	1.61*10^−3^	0.06	0.01
**BP**	rg						0.343*10–4	0.012	‒0.60*10^−4^	0.034	‒0.35*10^−4^	0.03	0.82**
	rp						3.431*10^−3^	1.26*10^−2^	‒6.04*10^−3^	6.8*10^−4^	‒3.35*10^−3^	8.2*10^−4^	‒0.13
**BW (g)**	rg							0.26*	0.29*	0.354*	0.13	‒0.68**	0.80**
	rp							0.24*	0.80**	1.10**	0.09	0.38*	3.42**
**SBD (cm)**	Rg								0.27*	0.07	0.02	‒0.53**	0.65**
	rp								0.07	‒0.28*	0.08	0.30*	0.55**
**GOT %**	rg									‒0.04	0.04	‒0.44**	0.75**
	rp									‒0.18	0.07	‒0.71**	-0.07
**SL (mm)**	rg										0.05	0.75**	0.91**
	rp										2.69*10^−3^	1.31**	2.68**
**FF (mic.)**	rg											0.02	-0.26
	rp											0.02	-0.93**
**FS (tpsi)**	rg												0.87**
	rp												1.82**

MBP = Monopodial branches per plant, MBL = monopodial branch length(cm), SBP = sympodial branches per plant, SBL = sympodial branch length, PH = plant height(cm), BP = bolls per plant, BW = boll weight(g), SBD = sympo-boll distance(cm), GOT = ginning out turn%, SL = staple length(mm), FF = fiber finesse (micronair), FS = fiber strength (tpsi), rg = genotypic correlation, rp = phenotypic correlation

** highly significant

* significant.

### Path analysis of yield components

Estimated genetic correlations were analyzed by partial regression equation to estimate direct and indirect effect of each individual trait understudy towards finally dependent trait like yield. Path analysis revealed logical and conclusive results of the study as monopodial branches per plant exerted a strong negative direct effect as (-0.54) but exhibited a strong positive indirect effect via monopodial branch length, plant height and bolls per plant as shown in (Table 3). Monopodial branch length exerted a positively strong direct effect was estimated as (1.15) on yield as key component and a moderate negative indirect effect via plant height (-0.4038) while other characters remained negligible as shown in (Table 3). Path analysis revealed a significantly strong negative direct effect of plant height was estimated as (-1.20), as compared it contributed quantitatively weak positive indirect effects via other traits understudy as shown in (Table 3). Bolls per plant exerted synchronously a strong positive direct effect on yield as (0.69) and indirectly by monopodial branches per plant. Sympo-boll distance exerted strong positive direct effect on yield as (0.81) with very negligible association or indirect effect via other plant traits As far as GOT% is concerned, path analysis revealed its moderate positive direct effect as yield component that impact a strong indirect effect via monopodial branches per plant as shown in (Table 3). Staple length exerted a positively strong direct effect on yield as (0.76) and very negligible contributions effected via other traits. Fiber finesse has been evaluated to exert a strong negative direct effect on yield and exhibited negligible effects indirectly via affecting other traits as shown in (Table 3). Finally, fiber strength has been estimated negligible direct effect on yield while it has been revealed an active component of yield via effecting strongly and positively correlated with other traits like monopodial branches per plant, sympodial branches per plant, and staple length synchronously and negatively effecting via other traits like boll weight sympo-boll distance and GOT% as shown in (Table 3).

**Table 3:** Direct (diagonal) and indirect (off-diagonal) genetic effect of yield components.

Variables	MBP	MBL (cm)	SBP	SBL (cm)	PH (cm)	BP	BW (g)	SBD (cm)	GOT %	SL (mm)	FF (mic.)	FS (tpsi)	rg
**MBP**	**‒0.54**	0.88	‒0.02	0.12	0.48	0.46	0.02	‒0.00	‒0.31	‒0.07	0.09	‒0.13	0.97
**MBL (cm)**	‒0.51	**1.15**	‒0.00	0.09	‒0.40	‒0.18	0.00	0.02	‒0.00	0.046	‒0.00	0.02	0.22
**SBP**	‒0.03	0.02	**‒0.42**	0.25	0.79	0.37	0.05	0.02	0.00	0.09	‒0.31	‒0.14	0.70
**SBL (cm)**	‒0.10	0.17	‒0.17	**0.63**	‒0.33	0.41	0.01	‒0.00	‒0.05	0.00	0.00	0.03	0.61
**PH (cm)**	0.21	0.38	0.28	0.17	**‒1.20**	0.06	‒0.00	0.00	‒0.01	0.029	‒0.00	0.01	‒0.05
**BP**	0.36	‒0.31	‒0.23	0.37	‒0.11	**0.69**	0.00	0.01	0.00	0.026	0.00	0.00	0.82
**BW (g)**	‒0.02	0.01	‒0.04	0.01	0.00	0.00	**0.54**	0.21	0.09	0.270	‒0.06	‒0.20	0.80
**SBD (cm)**	0.00	0.02	‒0.21	‒0.20	‒0.10	0.10	0.14	**0.81**	0.08	0.056	‒0.01	‒0.07	0.65
**GOT %**	0.54	‒0.00	‒0.00	‒0.20	0.04	0.00	0.16	0.22	**0.31**	‒0.03	‒0.12	‒0.15	0.75
**SL (mm)**	0.05	0.06	‒0.25	0.0006	‒0.04	0.02	0.19	0.05	‒0.01	**0.76**	‒0.02	0.09	0.91
**FF (mic)**	0.09	0.00	‒0.01	0.00	‒0.00	0.00	0.07	0.01	0.01	0.03	‒**0.50**	0.00	‒0.26
**FS (g per tax)**	0.56	0.18	0.47	0.18	‒0.29	0.22	‒0.47	‒0.44	‒0.23	0.57	‒0.01	**0.13**	0.87

## Discussion

Genetic variability in breeding material is a prime requisition of execution of an effective plant breeding program and selection strategies [18]. The breeding material that has been evaluated in this study acquired sufficient genetic variability for all the traits under study. We found strong positive correlation of monopodial branches per plant sympodial branches per plant, bolls per plant and boll weight and results of this study are in agreement with [21–24]. Our results partially deflected from [19] who reported significant and positive genetic correlation of staple length and fiber finesse to yield while we estimated significant and positive correlation estimates of fiber strength with seed cotton yield. Although, our results are in contrary with recently reported results of [25] they reported bolls per plant manifested highly strong direct positive effect on yield while micronaire value exhibited a moderate positive effect on yield. The other way, GOT% and uniformity ratio had strong negative direct effect following boll weight that had moderate negative direct effect on yield. The reported traits like bolls per plant, boll weight, lint yield per plant, GOT% and micronaire were suggested as robust indicators in selection of high yielding genotypes under saline conditions for improvement of seed cotton yield by [25].

A Path coefficient analysis is highly capable to simplify the exact interrelationship and contribution of each component effect on highly dependent variable like yield. Therefore, breeders are inclined to wisely focus on the set of components which shows high direct effect on yield and selection for those traits with positive moderate indirect effects to synchronize the selection efficiency. From path analysis and a careful review of the genetic correlations to harmonize the results, it is concluded that yield of cotton plant could be very effectively enhanced through direct selection of monopodial branch length, sympo-boll distance, staple length solely as these traits are independent of each other and not affecting antagonistically seed cotton yield via indirect effects. Secondly, an indirect selection is very effective for sympodial branch length via with bolls per plant. Conclusively, we suggest monopodial length, Sympo-boll distance and sympodial branch length as potential selection criterion for manipulation to improve the seed cotton yield.

In this study, we worked out the significance of three new genetic parameters via path analysis as yield components in aim to tentative manipulation of effective genetic parameters via selection in seed cotton yield improvement.

## Supporting information

S1 Data (XLSX)
